# Automatic Detection of Horner Syndrome by Using Facial Images

**DOI:** 10.1155/2022/8670350

**Published:** 2022-11-21

**Authors:** Jingyuan Fan, Bengang Qin, Fanbin Gu, Zhaoyang Wang, Xiaolin Liu, Qingtang Zhu, Jiantao Yang

**Affiliations:** ^1^Department of Microsurgery Orthopedic Trauma and Hand Surgery, The First Affiliated Hospital, Sun Yat-Sen University, Guangzhou 510080, China; ^2^Guangdong Province Engineering Laboratory for Soft Tissue Biofabrication, Guangzhou 510080, China; ^3^Guangdong Provincial Key Laboratory for Orthopedics and Traumatology, Guangzhou 510080, China

## Abstract

Horner syndrome is a clinical constellation that presents with miosis, ptosis, and facial anhidrosis. It is important as a warning sign of the damaged oculosympathetic chain, potentially with serious causes. However, the diagnosis of Horner syndrome is operator dependent and subjective. This study aims to present an objective method that can recognize Horner sign from facial photos and verify its accuracy. A total of 173 images were collected, annotated, and divided into training and testing groups. Two types of classifiers were trained (two-stage classifier and one-stage classifier). The two-stage method utilized the MediaPipe face mesh to estimate the coordinates of landmarks and generate facial geometric features accordingly. Then, ten machine learning classifiers were trained based on this. The one-stage classifier was trained based on one of the latest algorithms, YOLO v5. The performance of the classifier was evaluated by the diagnosis accuracy, sensitivity, and specificity. For the two-stage model, the MediaPipe successfully detected 92.2% of images in the testing group, and the Decision Tree Classifier presented the highest accuracy (0.790). The sensitivity and specificity of this classifier were 0.432 and 0.970, respectively. As for the one-stage classifier, the accuracy, sensitivity, and specificity were 0.65, 0.51, and 0.84, respectively. The results of this study proved the possibility of automatic detection of Horner syndrome from images. This tool could work as a second advisor for neurologists by reducing subjectivity and increasing accuracy in diagnosing Horner syndrome.

## 1. Introduction

Horner syndrome is a clinical constellation of signs and symptoms, typically consisting of the triad of miosis, ptosis, and facial anhidrosis. This syndrome was first comprehensively described by a Swiss ophthalmologist named Johann Friedrich Horner in 1869 [1]. Horner syndrome occurs when the sympathetic innervation of the eye is interrupted. Because of the long, circuitous anatomical pathway of the oculosympathetic efferent chain, the cause of Horner syndrome could be various. As the literature reported, Horner syndrome often does not have an identifiable cause, but 35%–60% cases of Horner syndrome were associated with neoplasms [2]. Considering the potentially life-threatening event, researchers recommended taking this syndrome as a “red flag” warning and deserving sufficient attention from all clinicians [3]. However, the diagnosis of Horner syndrome is often challenging due to the inconsistency of symptoms [3]. In addition, although the diagnosis could be improved by using clinical history, physical examination, and pharmacologic testing, it is still operator-dependent because of the subjectivity of pupillometry. Therefore, an objective diagnostic tool might be beneficial to clinicians.

Computer version methods have been widely applied to process medical images for providing object predictions in these years. Recent studies have achieved outstanding accuracy in the classification of skin lesions from dermoscopic images [4], malignancy detection on mammography [5], the diagnosis of acute lymphoblastic leukemia [6], the detection of retinopathy in retinal fundus photographs [7], as well as the detection of COVID-19 from CT scans [8, 9] and X-ray images [10]. However, this technique is rarely used to detect clinical signs, such as the Horner sign.

This study presents an objective method for detecting Horner syndrome from face images. Here, we proposed two methods for this task: the two-stage and the one-stage methods. The two-stage method contained two steps: the first step was landmark extraction by MediaPipe face mesh [11], and the second step was the construction of conventional machine learning classifiers. The one-stage method transferred Horner syndrome recognition into an object detection task that can directly recognize Horner syndrome from facial photos. Here, we utilized one of the latest and most powerful algorithms in this field, YOLO v5 [12], which can carry out regional proposal and classification simultaneously for this task. Our method may provide a possibility for the detection of Horner syndrome. These classifiers could act as reliable assistants for neurologists in the near future.

## 2. Materials and Methods

### 2.1. Data Sources

Our dataset was acquired from the image dataset of patients with brachial plexus injury in our department. The acquisition was performed following relevant regulations and proved by the ethics committee of our institution. Images that fulfilled the following criteria were as follows: (1) images containing both eyes and at least 2/3 face of the subject; (2) images shot in sufficient light and had an adequate resolution for pupil observation. The exclusion criteria were as follows: (1) the face in the image had apparent tilt or rotation; (2) images contained more than one person. The whole process of this study is illustrated by a flow chart (Figure 1).

### 2.2. Annotation Procedure

Image annotation greatly influences the quality of the dataset, which could impact the accuracy of the final model. For that, we had two experts with 14 and 26 years of experience, respectively, to label the data together. Images and necessary information, including case history and EMG and MRI scan results, were provided to them to get a precise diagnosis. The label was obtained on the consensus of the two experts. In cases with conflict, they thoroughly re-evaluated and discussed to reach a final diagnosis. The image would be excluded if the agreement cannot be reached after reviewing all available information.

### 2.3. Dataset Splitting

The images in the dataset were randomly split into two parts: the training set and the testing set. The splitting scheme was 75/25. The training set was used to train and validate the model, while the testing set was used to evaluate the model's performance.

### 2.4. Data Augmentation

To overcome the issue of insufficient training data and increase the robustness of the model, we applied data augmentation by using the albumentations library [13]. Images were expanded by ten times after adding Gaussian and multiplicative noise, RGB shifting, contract/brightness/scale changes, flipping, and cropping.

### 2.5. Model Construction

#### 2.5.1. Two-Stage Detection Classifier

The two-stage detection classifier contained two main steps. The first step was extracting facial landmarks and the second was the construction of machine learning classifiers using the extracted features. In this work, we used the facial landmark detector from the MediaPipe library [11] to generate landmarks on the face images. This model is able to output the 3D position of 468 face landmarks from an image, containing information on various facial areas such as the cheeks, forehead, mouth, and eyes. Considering Horner signs mainly influence the appearance of the eyes and the periocular regions, we selected 32 landmarks to generate geometric features for the classifier. To represent the geometric features efficiently, we converted the coordinates of landmarks to distances between points and angles between edges. A total of 22 (11 for each side) parameters were selected to characterize the geometric features of the interest area (shown in Figure 2). Each parameter was estimated in two manners (the MediaPipe face mesh could estimate the coordinate of landmarks in both 2-dimension and 3-dimension manners). Then, to eliminate individual differences, we generated ratios of these parameters between the left and right sides. All the ratios were calculated by dividing the smaller value into the larger value to prevent the effect caused by the side.

After data standardization, we performed feature decomposition using principal component analysis (PCA). Then, the features were fed to classifiers. In this work, logistic regression, K-neighbors, decision tree, support vector machine (SVM), Bernoulli naïve Bayes, Random Forest, GradinetBoosting, AdaBoost, Light GBM, and XgBoost were used for classification. The grid-search method [14] was used to identify the optimal hyperparameters and structure of the classifier. In addition, the five-fold cross-validation was also employed to assess the combination of hyperparameters to avoid overfitting. In this procedure, the training set was further split into five subsets. Four subsets were used to train the classifier, while the remaining one was used to validate the accuracy. The optimal configurations in this stage were applied in the testing set.

#### 2.5.2. One-Stage Detection Classifier

YOLO (you only look once) family is one of the most powerful and fastest deep learning object detection algorithms. Unlike the other object detection techniques that send multiple patches to the classifier, the YOLOs send the whole image to a single convolutional neural network (CNN). This CNN predicted the bounding box, as well as the class possibilities at the same time. It was first presented by Redmon et al. in 2016 [15]. In this study, we utilized the latest version, YOLO v5 [12], to detect Horner syndrome. The region of interest (ROI) was the portion of the image containing the eyes and periocular areas. Since the data were insufficient in this work, we chose to freeze the convolution layers and retrain the fully connected layer rather than start from scratch. The pretraining weights (yolov5s) were used as the initial weights. The YOLO classifier was trained through 2000 epochs, with a batch size of 32, a learning rate of 0.01, a weight decay of 0.005, and a momentum of 0.937.

### 2.6. Model Evaluation

The performance of the classifier was evaluated by assessing the diagnosis accuracy, sensitivity, and specificity. The receiver operating characteristic (ROC) curve was used to illustrate the capacity of two-stage classifiers. The precision-recall curve with mean average precision at IoU (Intersection-Over-Union) = 0.5 (mAP@0.5) was used to show the performance of the one-stage classifier. In addition, confusion matrices were employed to present whether the predictions of classifiers were discordant with the gold standard.

### 2.7. Statistical Analysis

Experiments were performed on three Intel(R) Xeon(R) CPUs with 8 GB RAM and a NVIDIA RTX 3090 GPU with 24 GB RAM. Python 3.7 was used as the development environment. OpenCV was used for image preprocessing, and albumentations was used for data augmentation. The MediaPipe library was used for facial landmarks extraction. Scikit-learn was used for constructing the machine learning classifiers and compute the evaluation metrics. NumPy, Pandas, OS, and Matplotlib were also used in this procedure.

## 3. Results

### 3.1. Clinical Characteristics

In total, 173 images of patients were collected in our dataset. Sixty-nine images of patients were diagnosed with Horner (+), while the remaining ones were Horner (−). The included images were split into training and testing sets, then the data augmentation was performed. The training and testing sets had 1350 (510 positives and 840 negatives) and 380 (140 positives and 240 negatives) images, respectively. The resolution of included images ranged from 455*∗*837 to 2848*∗*4288.

### 3.2. Descriptive Statistics of Extracted Features

With a minimum detection confidence of 0.7, the MediaPipe face mesh failed to detect human faces in 40 and 27 images in the training and testing sets. Therefore, only 1310 images (478 positives and 832 negatives) were entered into feature extraction, and 353 images (118 positives and 235 negatives) were used for model evaluation. The detection rate was 97.03% and 92.9%, respectively. Then, the ratios of selected geometric features were calculated (shown in Figure 2). The distribution of data in training and testing sets is summarized in Table 1. Principal component analysis identified 11 components that explained 98.22 percent of the variance between the positive and negative cases (Figure 3(a)). The composition of each principal component is presented in Figure 3(b). The optimal hyperparameters of each classifier were identified by the grid-search method and shown in Table 2.

All the features were presented as ratio, and the generation process is shown in the methods' part. sd: standard deviation.

### 3.3. Model Performance

#### 3.3.1. Two-Stage Classifier

The performances of the machine learning classifiers are sorted from high to low according to the prediction accuracy (shown in Table 3). The decision tree classifier held the highest accuracy (0.790), followed by KNN, XgBoost, gradient boost classifier, logistic regression, support vector classifier, LGBM, random forest classifier, AdaBoost classifier, and Bernoulli NB. The sensitivity, specificity, positive predictive value, and negative predictive value are also presented in Table 3. Confusion matrices in Figure 3(c) present the number of true positive, false positive, true negative, and false negative. In addition, the visual comparison between the classifier was also generated by using the receiver operating characteristic curve (Figure 3(d)). The gradient boost classifier produced the highest AUC (0.830), while the decision tree classifier produced the lowest (0.628).

#### 3.3.2. One-Stage Classifier

The performance of the one-stage classifier was summarized in Figure 4(a), which shows the change of accuracy and losses during the training process. The accuracy, sensitivity, and specificity of the classifier were 0.65, 0.51, and 0.84, respectively. The classification performance of this classifier was also presented by the confusion matrix (Figure 4(b)) and the precision-recall curve (Figure 4(c)). The average precision of negative, positive, and all classes were 0.702, 0.838, and 0.770, respectively.

## 4. Discussion

This work presented two approaches for automatic Horner syndrome detection from facial images. The two-stage method integrated an automatic face landmark generator MediaPipe with machine learning classifiers. The one-stage method utilized an object detection algorithm, YOLO v5. Both methods achieved adequate accuracy in this task. To the best of our knowledge, this is the first study trying to detect Horner syndrome automatically, and the results proved that the computer output could act as a second adviser for neurologists and contribute to doctors before making the final decisions.

Horner syndrome arises from a lesion or a disruption along the oculosympathetic efferent chain, which a variety of etiologies can cause. The typical triad of Horner syndrome is ipsilateral ptosis, pupillary miosis, and facial anhidrosis [16]. However, all three symptoms are not consistently present and are always subtle. According to a report of 318 patients, less than 2% of patients presented with anhidrosis, and ptosis was recorded in only 34% of patients [17]. Although the occurrence rate of miosis was relatively high (91%) [17], the observation of it is significantly impacted by light [18]. Usually, miosis is more apparent in the dark, and the so called “dilation lag” is only apparent within the first few seconds [18, 19]. The actual degree of miosis could also be impacted by several factors including the resting size of pupil, alertness of the patients, and sympathetic drive [18]. Therefore, the presence of Horner syndrome can easily be overlooked in clinical practice. Although ptosis and miosis of Horner syndrome are not likely to cause any functional disturbance, the detection of Horner syndrome is still critical, as its cause can be very threatening or sometimes lethal. Previous studies have indicated that Horner syndrome should be considered a “red flag” warning, and thus, the recognition and evaluation are important to all clinicians [3].

Typically, the diagnosis of Horner syndrome was confirmed by several pharmacological agents such as cocaine, apraclonidine, and hydroxyamphetamine. However, the use of these agents has many drawbacks. First, some of the agents are controlled drugs and rarely available. It is impractical to use them in general departments. Second, the construction of pharmacological tests and the pupillometry after drug use require the experience of the operator, and therefore, it is hard to normalize and generalize. Third, the sensitivity of pharmacological tests needs further validation because there are several reports of false negative cases [20, 21]. In addition, the results of these tests could be influenced by the time from the onset of damage [22, 23], as well as the use of other drugs [19]. Therefore, a diagnostic tool other than drugs may benefit clinical practice.

In this study, we present a method to detect Horner syndrome from digital images. Actually, the image is the most commonly used method for the recording of Horner signs previously. Our method may provide a new way to diagnose without additional burdens. The two types of classifiers all showed adequate accuracy. For the two-stage method, we used MediaPipe for the face landmark extraction and trained machine learning models according to the coordinates of landmarks. This cooperation has been utilized in several previous studies. Siam et al. [24] used facial landmarks to generate geometrical features for human emotion classification and demonstrated superior performance. In the report of Gomez et al. [25], they analyzed the evoked facial gestures in patients with 'Parkinson's Disease from the video of patients and indicated that the detection rate significantly improved (from 75.00% to 88.46%) by using the 17 facial features derived from the landmark detection algorithm. In addition, similar attempts have also been applied in the assessment of cerebral palsy [26], pose evaluation in sports [27, 28], and human activity recognition [29]. The combination of pose estimation methods and machine learning classifiers presented superior performances in these works. In our study, we utilized landmarks around the eyes to generate parameters for this task because Horner syndrome mainly influences the geometrical features around the eyes. However, as mentioned above, ptosis is not consistently present in Horner (+) patients [17], and it is common to observe asymmetry in eyes among healthy individuals. Therefore, it is not hard to understand the relatively high specificity and low sensitivity of these models.

As for the one-stage classifier, the YOLO v5 is the latest version of the most powerful and fastest object detection algorithms. The YOLO family has been utilized in many medical tasks including the detection of lung nodules [30], breast abnormalities [31], and lymphocytes [32] and achieved high accuracy. However, in this paper, the predictive accuracy was slightly lower than the two-stage classifiers. We assumed that it was due to the insufficient data volume, although we have used data augmentation and transfer learning technology. At present, data deficiency in medical imaging is a common problem for all researchers. This is extremely obvious in our task because the incidence of Horner syndrome is not so high, and there was no existing database of this syndrome. Future studies with more images are needed to develop this model.

The lack of powerful computers is an inevitable problem in most clinical settings [33]. Therefore, for medical use, the running speed of the model is just as important as its accuracy. In this study, both deep learning models are characterized by fast running speed and well performance [11, 34]. The MediaPipe face mesh (BlazeFace) [11] showed super-real-time performance (200–1000+ frames per second) on mobile devices and achieved an average precision (AP) of 98.61% in the testing dataset. Similarly, YOLO v5 was presented as an efficient and powerful object detection model [34] and achieved state-of-the-art performance with a speed of 140 frames per second on Tesla P100, which performs twice faster as the previous version [35]. Without the requirement of excessive computational power support, these methods are more suitable for application in real clinical settings. As for the model performance in this study, the specificities of classifiers were much higher than the sensitivities. This characteristic indicates that these proposed models can help rule out patients with oculosympathetic pathway problems. These detectors can curtail the necessity for examination for all patients, thereby saving time and resources. In addition, the automatic detection can also benefit primary hospitals, where there are no available experts to rule out those high-risk patients.

This study also has some limitations. Firstly, due to the rarity of Horner (+) patients, the study only involved a limited number of samples. Future studies with larger sample sizes may help to enhance robustness and improve the accuracy of this method. Secondly, all the diagnoses of Horner syndrome were derived from patients with brachial plexus injury. The diverse prevalence in different diseases might affect the sensitivity and specificity of detectors, which could also impact the potential generalizability of the results. Thirdly, although facial images are the most convenient and commonly used method for recording Horner syndrome, videos can provide dynamic information and have great potential to achieve better results. To solve these problems, we will establish the Horner syndrome database with various patients caused by different primary diseases. In addition, we will also attempt to investigate the possibility and accuracy of video detection.

## 5. Conclusions

In summary, we proposed two pipelines to detect Horner syndrome from facial images and evaluated their performance. Both the methods presented adequate accuracy compared with human experts. Our results have proved the possibility of automatic Horner detection, which could work as a second advisor to rule out high-threatening patients.

## Figures and Tables

**Figure 1:** The process of model construction and evaluation.

**Figure 2:** Examples of the facial landmarks generated by MediaPipe and the parameters used to characterize the face.

**Figure 3:** The performance of the two-stage classifier (a) the process of the principal component analysis (PCA); (b) the composition of each principal component; (c) ROC curves of the ten included machine learning classifiers; (d) confusion matrices of the ten included machine learning classifiers.

**Figure 4:** The performance of the one-stage classifier (a) the training process of the YOLO v5-based classifier; (b) the confusion matrices of the one-stage classifier; (c) the precision-recall curve of the one-stage classifier.

**Table 1:** Summary of the dataset distribution.

Features (ratio)	Training set ($\bar{x}$ ± sd)			Testing set ($\bar{x}$ ± sd)		
	Positive	Negative	Whole	Positive	Negative	Whole
Distance_1	1.164 ± 0.137	1.081 ± 0.137	1.111 ± 0.103	1.169 ± 0.085	1.073 ± 0.060	1.105 ± 0.083
Distance_2	1.154 ± 0.129	1.078 ± 0.129	1.105 ± 0.098	1.165 ± 0.095	1.070 ± 0.053	1.102 ± 0.083
Distance_3	1.148 ± 0.124	1.077 ± 0.124	1.103 ± 0.096	1.160 ± 0.099	1.072 ± 0.050	1.102 ± 0.082
Distance_1_3d	1.159 ± 0.131	1.079 ± 0.131	1.108 ± 0.100	1.167 ± 0.084	1.071 ± 0.058	1.103 ± 0.081
Distance_2_3d	1.150 ± 0.124	1.076 ± 0.124	1.103 ± 0.095	1.164 ± 0.094	1.069 ± 0.052	1.101 ± 0.082
Distance_3_3d	1.144 ± 0.120	1.075 ± 0.120	1.100 ± 0.093	1.159 ± 0.097	1.070 ± 0.048	1.100 ± 0.080
Distance_4	1.112 ± 0.100	1.117 ± 0.100	1.115 ± 0.092	1.079 ± 0.051	1.065 ± 0.043	1.069 ± 0.046
Distance_5	1.079 ± 0.069	1.068 ± 0.069	1.072 ± 0.059	1.096 ± 0.073	1.062 ± 0.041	1.074 ± 0.057
Distance_6	1.112 ± 0.102	1.094 ± 0.102	1.100 ± 0.088	1.034 ± 0.024	1.032 ± 0.023	1.033 ± 0.023
Distance_7	1.046 ± 0.040	1.044 ± 0.040	1.045 ± 0.036	1.051 ± 0.039	1.041 ± 0.029	1.044 ± 0.033
Distance_4_3d	1.065 ± 0.049	1.072 ± 0.049	1.070 ± 0.050	1.128 ± 0.097	1.096 ± 0.068	1.107 ± 0.080
Distance_5_3d	1.068 ± 0.058	1.057 ± 0.058	1.061 ± 0.049	1.107 ± 0.081	1.075 ± 0.052	1.085 ± 0.064
Distance_6_3d	1.034 ± 0.026	1.033 ± 0.026	1.034 ± 0.025	1.153 ± 0.117	1.087 ± 0.062	1.109 ± 0.090
Distance_7_3d	1.045 ± 0.039	1.043 ± 0.039	1.044 ± 0.035	1.052 ± 0.040	1.042 ± 0.029	1.046 ± 0.033
Angle_1	1.109 ± 0.086	1.077 ± 0.086	1.089 ± 0.074	1.109 ± 0.104	1.063 ± 0.051	1.079 ± 0.076
Angle_2	1.130 ± 0.109	1.071 ± 0.109	1.092 ± 0.087	1.144 ± 0.110	1.078 ± 0.053	1.100 ± 0.083
Angle_3	1.142 ± 0.154	1.098 ± 0.154	1.114 ± 0.110	1.140 ± 0.075	1.063 ± 0.051	1.089 ± 0.071
Angle_4	1.138 ± 0.125	1.086 ± 0.125	1.105 ± 0.095	1.160 ± 0.099	1.066 ± 0.045	1.097 ± 0.082
Angle_1_3d	1.110 ± 0.091	1.083 ± 0.091	1.093 ± 0.077	1.100 ± 0.097	1.060 ± 0.046	1.073 ± 0.070
Angle_2_3d	1.131 ± 0.111	1.077 ± 0.111	1.096 ± 0.088	1.144 ± 0.101	1.075 ± 0.053	1.098 ± 0.079
Angle_3_3d	1.135 ± 0.110	1.068 ± 0.110	1.093 ± 0.086	1.159 ± 0.125	1.070 ± 0.049	1.100 ± 0.093
Angle_4_3d	1.131 ± 0.109	1.068 ± 0.109	1.091 ± 0.085	1.169 ± 0.138	1.069 ± 0.050	1.102 ± 0.101

**Table 2:** The optimal hyperparameters of machine learning classifiers.

Models	Hyperparameters
Decision tree	{Max depth: 3, max leaf nodes: 4, min samples leaf: 5, and min samples split: 165}
K-neighbors	{*n* neighbors: 30}
XgBoost	{Learning rate: 0.01, max depth: 3, *n* estimators: 100, and subsample: 0.3}
Gradient boosting	{Learning rate: 0.05, max depth: 1, *n* estimators: 30, and subsample: 0.3}
Logistic regression	{*C*: 0.1, l1 ratio: 0.01, max iter: 10000, and solver: Liblinear}
Support vector classifier	{*C*: 0.5, degree: 1, kernel: “Linear”}
Light GBM	{Learning rate: 0.2, max depth: 3, *n* estimators: 15, and subsample: 0.3}
Random forest	{Max depth = 2, max features = 3, and *n* estimators = 5}
AdaBoost	{Learning rate: 0.2, *n* estimators: 20}
Bernoulli naïve bayes	{Default}

**Table 3:** The performances of machine learning classifiers.

Classifiers	Sen	Spe	PPV	NPV	Acc
Decision tree	0.432	0.970	0.879	0.773	0.790
K-neighbors	0.483	0.940	0.803	0.784	0.788
XgBoost	0.39	0.983	0.920	0.762	0.785
Gradient boosting	0.373	0.987	0.936	0.758	0.782
Logistic regression	0.364	0.987	0.935	0.756	0.779
Support vector classifier	0.356	0.987	0.933	0.753	0.776
Light GBM	0.322	0.979	0.884	0.742	0.759
Random forest	0.254	0.996	0.968	0.727	0.748
AdaBoost	0.237	0.996	0.966	0.722	0.742
Bernoulli naïve Bayes	0.331	0.902	0.629	0.729	0.711

Sen: sensitivity, Spe: specificity, PPV: positive predictive value, NPV: negative predictive value, and Acc: accuracy.

## Data Availability

The raw data required to reproduce these findings cannot be shared at this time as the data also form a part of an ongoing study. The processed data are available upon request by contact with the corresponding author.
